# Mir-204 Regulates LPS-Induced A549 Cell Damage by Targeting FOXK2

**DOI:** 10.1155/2021/7404671

**Published:** 2021-11-30

**Authors:** Shufen Li, Lifen Zhao, Xujiong Li, Gaiping Shang, Lijing Gao, Zhuohui Song, Ting Li

**Affiliations:** ^1^Department of Physiology, Changzhi Medical College, Changzhi, Shanxi 046000, China; ^2^Department of Respiratory and Critical Care Medicine, Shanxi Academy of Hospital Sciences, Taiyuan, Shanxi 046000, China; ^3^Department of Respiratory and Critical Care Medicine, Shanxi Bethune Hospital, Taiyuan, Shanxi 046000, China

## Abstract

**Objective:**

To assess whether miR-204 and HA affect A549 cell injury induced by lipopolysaccharide. *Material and Methods*. A549 cells were treated with hirsutanol A, and cell damage was induced by LPS followed by analysis of cell proliferation by CCK-8, cell apoptosis by flow cytometry, apoptosis-related protein expression by western blot, downstream target of miR-20 by dual-luciferase reporter gene, and inflammatory factors by ELISA and PCR.

**Results:**

LPS can significantly inhibit the viability of A549 cells, induce cell apoptosis, and promote the release of IL-6, IL-1*β*, and TNF-*α*, while HA pretreatment can target FOXK2 by upregulating miR-204 levels, thereby alleviating apoptosis and promoting cell viability and at the same time inhibiting the release of inflammatory factors by inhibiting the activation of NF-*κ*B.

**Conclusions:**

miR-204 participates in the protection of HA acute lung injury by targeting FOXK2.

## 1. Introduction

Acute lung injury (ALI) has a high morbidity and mortality [1–3]. ALI is featured as destruction of the alveolar-capillary membrane barrier leading to inflammation and subsequent lung dysfunction [4, 5]. Therefore, inhibiting inflammation may be critical to ALI treatment. Hirsutanol A (HA) has a strong cytotoxic effect as a sessile mushroom compound. Studies have found that HA can induce tumor cell apoptosis by upregulating cleaved-caspase-3, but it is rarely reported in ALI and ARDS [6, 7].

miRNA dysregulation involves in inflammatory diseases. Recent studies demonstrated that [8, 9] miR-204 participates in sepsis. For example, miR-204 can protect early sepsis by inhibiting the release of proinflammatory factors through GSKJ4, and miR-204 can also inhibit the NF-*κ*B pathway and FOXK2 to downregulate miR-21, thereby improving the occurrence of sepsis, but its effect on sepsis-induced ALI is not yet known. According to reports [10, 11], excessive oxidative stress and inflammation play a crucial role in the pathogenesis of ALI. Nrf-2 is a pleiotropic protein that inhibits the transcriptional activation of its downstream target NF-*κ*B by acting on antioxidant response elements and ultimately regulates the expression of a series of antioxidants and other genes [12]. Recent studies have shown that [13, 14] miR-204 is a new regulator of innate immune response, which can significantly improve the survival rate of LPS-induced sepsis by preventing NF-*κ*B-mediated inflammation. This study established an acute lung injury model induced by lipopolysaccharide and explored the specific mechanism of miR-204 in lung injury induced by lipopolysaccharide and the specific mechanism of HA.

## 2. Materials and Methods

### 2.1. Cell Culture and Processing

A549 was purchased from Celera Stem Cell Technology Co., Ltd. (China) and was cultured in DMEM medium (Celera Stem Cell Technology Co., Ltd., China). After culturing the cells in 96-well plates for 24 hours, the treatment group was pretreated with HA (1.25, 2.5, 5, and 10 *μ*M) for 15 minutes, and then, LPS (20 *μ*g/mL, Sartorius Bioreagent, Germany) was added to each well for 12 hours. To create a cell injury model, the control group was treated with dimethyl sulfoxide (DMSO).

### 2.2. CCK-8 Assay

Cells (1000 cells/well) in a 96-well plate were collected after treatment for 24 hours. Based on kit instructions, 10 *µ*L CCK-8 solution was added to measure the absorbance at 450 nm (Annolun Biotechnology Co., Ltd., China) with a microplate reader to evaluate cell viability.

### 2.3. Analysis of Cell Apoptosis

The cells (1000 cells/well) were cultured in 96-well plates and were harvested after 24 hours of different treatments. Based on kit instructions, they were washed twice with 1x phosphate buffered saline (Virencer Bioreagent Co., Ltd., China). Based on the manufacturer's instructions (Chengdu Lingdong Biotechnology Co., Ltd., China), we used the FITC/PI cell apoptosis detection kit (Jianglan Pure Biological Reagent Co., Ltd., China) to detect cell apoptosis, incubated in the dark for 15 minutes, and then, performed FACScan flow Cytometry (Boaosen Biotechnology Co., Ltd., China) to analyze cell apoptosis [15].

### 2.4. ELISA

IL-1*β*, IL-6, and TNF-*α* in cell supernatant (Jianglan Pure Biological Reagent Co., Ltd., China) was measured by using the ELISA kit based on kit instructions.

### 2.5. Cell Transfection

When the cells grow to the logarithmic growth phase, according to the manufacturer's recommendations, we used pDONR223-FOXK2 (Hengdailau Biotechnology Co., Ltd., China) with an inserted stop codon to construct the FOXK2 overexpression vector and named it p-FOXK2. According to the manufacturer's instructions, we used Lipofectamine 2000 (Hengdai Lao Biotechnology Co., Ltd., China) for transfection. miR-204 mimic and corresponding negative control (NC) were from Nantong Yishi Biotechnology Co., Ltd. (China).

### 2.6. qPCR

According to the manufacturer's recommendations, Trizol (Weirun Sairun Biological Reagent Co., Ltd., China) extracted total cellular RNA followed by cDNA synthesis using a one-step miRNA RT kit (Golden Times Biotechnology Co., Ltd., China). Then, qPCR was performed using the ABI Prism 7500 detection system with a TaqMan multiplex qPCR master mix (Botuo Biotechnology Co., Ltd., China) to detect mRNA and miNRA levels. GAPDH was selected as a reference. Gene level was analyzed using the 2−△△ct method [16].

### 2.7. Western Blot

RIPA lysate containing protease inhibitors (Chengdu Lingdong Biotechnology Co., Ltd., China) extracted total cell protein which was quantified by using a BCA kit (Chengdu Lingdong Biotechnology Co., Ltd., China) followed by separation on 12% SDS-PAGE for western blot using antibodies against Bax (1 : 2000, Serera Stem Cell Technology Co., Ltd., China), Bcl-2 (1 : 2000, Sartorius Bioreagents, Germany), caspase-3 (1 : 1000, Lihan Biotechnology Co., Ltd., China), I-*κ*B (1 : 2500, Mao Kang Biotechnology Co., Ltd., China), and GAPDH (1 : 5000, Mao Kang Biotechnology Co., Ltd., China).

### 2.8. Luciferase Reporter Gene

The FOXK2 3′UTR or mutant was cloned into a pMIR-Report vector (Ruikai Stem Cell Biotechnology Co., Ltd., China), named Luc-FOXK2-wt or Luc-FOXK2-mut. A549 cells were cotransfected with miR-145 mimic or negative control and Luc-FOXK2-wt or Luc-FOXK2-mut for 72 hours followed by analysis of luciferase activity checked by using a luminometer (Boaosen Biotechnology Co., Ltd., China).

### 2.9. Statistical Processing

The data were processed by GraphPad Prism 9 software and displayed as mean ± SD and evaluated by ANOVA or Student's *t*-test. *P* < 0.05 indicated significance.

## 3. Results

### 3.1. HA Alleviates LPS-Induced Apoptosis and Cell Viability Inhibition

LPS can significantly inhibit cell viability and induce cell apoptosis (Figures 1(b) and 1(c)); HA alone has no significant effect on cell viability (Figure 1(a)); compared with the LPS group, HA treatment can significantly inhibit cell apoptosis and promote cell proliferation (Figures 1(b) and 1(c)).

Western blot analysis showed that, after LPS treatment, apoptosis-related protein was significantly upregulated, while antiapoptotic protein was significantly downregulated. HA pretreatment can effectively inhibit the expression of apoptotic protein and upregulate Bcl-2 (Figure 1(d)). Further ELISA testing showed that inflammatory factors in the cell supernatant of the LPS group were significantly increased, which were inhibited by HA (Figures 1(e) and 1(f)).

### 3.2. HA Inhibits LPS-Induced Apoptosis by Regulating miR-204

PCR analysis showed that, after treatment with LPS, miR-204 was significantly downregulated, which was upregulated by HA (Figure 2(a)). Meanwhile, miR-204 inhibitor can effectively inhibit miR-204 level (Figure 2(b)).

LPS treatment can significantly inhibit cell viability and promote cell apoptosis, which were reversed by HA. After miR-204 inhibitor transfection, cell viability was significantly reduced and apoptosis was significantly increased (Figures 2(c) and 2(d)); protein immunoblot analysis showed that HA pretreatment can effectively reverse LPS-induced apoptosis protein expression. After miR-204 inhibitor transfection, apoptotic protein was significantly upregulated while antiapoptotic protein was downregulated (Figure 2(e)). It is suggested that HA can alleviate LPS-induced apoptosis and cell viability inhibition by regulating miR-204. Further ELISA tests showed that HA pretreatment can effectively reverse the release of inflammatory factors induced by LPS, while miR-204 inhibitor can reverse the anti-inflammatory effect of HA and upregulate inflammatory factors (Figures 2(f) and 2(g)), indicating that HA can regulate miR-204 to alleviate the inflammatory environment induced by LPS.

### 3.3. miR-204 Targets and Regulates FOXK2

Predictions by TargetScan show that FOXK2 3 in the UTR region can bind miR-204 (Figure 3(a)), and further dual-luciferase reporter gene detection shows that compared with FOXK2-WT, miR-204 mimic treatment can effectively inhibit fluorescence. Compared with FOXK2-MUT, miR-204 mimic treatment had no significant effect (Figure 3(b)), indicating that miR-204 is a target of FOXK2.

### 3.4. miR-204 Participates in HA Alleviating LPS-Induced Lung Injury through Targeted Regulation of FOXK2

FOXK2 expression in A549 cells was significantly increased after FOXK2 plasmid transfection (Figure 4(a)). HA pretreatment can effectively reverse cell viability and apoptosis induced by LPS. When cells are transfected with miR-204 inhibitor, cell viability is significantly reduced and apoptosis is significantly increased. The viability of A549 cells was significantly restored after FOXK2 plasmid infection, and cell apoptosis was significantly reduced (Figures 4(b) and 4(c)).

Western blot analysis showed that, after miR-204 inhibitor treatment, the apoptotic protein increased and the antiapoptotic protein level was downregulated (Figure 4(d)). Further ELISA tests showed that release of inflammatory factors was significantly increased after transfection with miR-204 inhibitor and cotransfection with FOXK2 plasmids inhibited the upregulation of inflammatory factors induced by miR-204 inhibitor (Figures 4(e) and 4(f)).

### 3.5. Silencing miR-204 Inhibits the NF-*κ*B Pathway by Regulating FOXK2

LPS can significantly promote NF-*κ*B activation and HA treatment can inhibit the activation of the NF-*κ*B pathway induced by LPS. After transfection with miR-204 inhibitor, the activation of NF-*κ*B inhibited by HA is obvious. However, NF-*κ*B activation promoted by miR-204 inhibitor was significantly inhibited after cotransfection of FOXK2 plasmid, indicating that silencing miR-204 participates in the inhibition of the LPS-induced NF-*κ*B pathway by regulating FOXK2 (Figure 5).

## 4. Discussion

Sepsis is a main cause of death in patients with trauma, burns, and severe surgery [17]. Among them, acute lung injury caused by sepsis appears first [18]. The results of this study showed that, in the LPS-induced in vitro model of ALI, miR-204 was significantly downregulated. The downregulated miR-204 activates the NF-*κ*B pathway by targeting FOXK2, promotes the release of inflammatory factors, and induces A549 cell apoptosis, and HA can exert ALI protection by upregulating miR-204.

In order to study the molecular mechanism of human ALI, the endotoxin model induced by LPS was used. We showed that, after treatment with LPS for 24 hours, cell apoptosis was significantly increased and cell viability was significantly inhibited, while after HA pretreatment, the apoptosis of A549 cells was significantly reduced and cell viability was significantly increased. It has been reported [19, 20] that the downregulation of miR-204 can induce type II epithelial cell apoptosis in ALI. In addition, the literature pointed out [21] that miR-204 overexpression in the lung can reduce lipopolysaccharide-induced permeability index and inhibit the release of inflammatory cytokines in lung histology. The recent literature pointed out [22] that miR-204 can upregulate epithelial sodium channels (ENaCs), a critical molecule for alveolar fluid clearance. We showed significantly downregulated miR-204 in the lung injury model along with increased apoptotic protein and decreased antiapoptotic protein, reduced cell viability, and promoted cell apoptosis. When HA is used, the transcription level of miR-204 is significantly increased, and LPS-induced apoptosis and cell viability inhibition are significantly reversed. After further transfection with miR-204 inhibitor, the protective effect of HA is significantly reversed. FOXK2 is a target for miR-204 to exert teratogenicity and cytotoxicity, and it plays a vital role in cellular processes [23]. Therefore, abnormal expression of FOXK2 leads to the occurrence of many diseases and their development. According to reports [24], FOXK2 can inhibit NF-*κ*B activation, and NF-*κ*B regulates inflammation and oxidative stress and is involved in various inflammations. In the development of sexual diseases, recent the work in [25] pointed out that NF-*κ*B activation may cause release of inflammatory mediators, thereby enhancing lung inflammation and inducing ALI. Therefore, we hypothesized that FOXK2 may be involved in the biological role of miR-204 in the development of ALI. We confirm that miR-204 in A549 cells can target 3, UTR of FOXK2. When treated with miR-204 inhibitor, the inhibitory effect of HA and the protective effect of A549 were reversed. After further cotransfection with FOXK2, the viability of A549 cells was significantly restored, apoptosis was reduced, and the level of inflammatory factors released decreased. The redox state of cells regulates NF-*κ*B activation induced by LPS. For example, Nrf-2 regulates NF-*κ*B activation by regulating cellular antioxidants to maintain the redox state of the cell, and the increased activation of NF-*κ*B promotes inflammation caused by LPS. We found that LPS significantly promoted the release of inflammatory factors and activated the NF-*κ*B pathway, while HA or FOXK2 vector cotransfection reversed FPS or miR-204 inhibitor-induced NF-*κ*B activation, thereby inhibiting inflammatory factor release.

In summary, HA can significantly alleviate the damage of A549 cells induced by LPS by upregulating miR-204. miR-204 involves in HA's effect on lung injury. FOXK2 was a target of miR-204. The protective effect of HA on A549 cells may be achieved by regulating miR-204 and then regulating FOXK2. The results of this article provide a theoretical basis for targeted therapy of acute lung injury. However, this study also has certain limitations. For example, in vivo experiments were not performed, and oxidative stress indicators in acute lung injury were not tested. In addition, Nrf-2, the upstream of the inflammatory factor-related pathway, was not tested.

## Figures and Tables

**Figure 1:** HA alleviates LPS-induced lung injury. (a) The effect of HA treatment on cell viability; (b) HA treatment alleviated the decrease in cell viability; (c) HA alleviated cell apoptosis induced by LPS; (d) HA alleviated the apoptosis of A549 cells LPS-induced upregulation of the expression of apoptosis-related proteins; (e) HA alleviated the increase in inflammation-related factors; and (f) HA alleviated the increase in inflammation-related factors. Compared with the LPS group, ^*∗*^*P* < 0.05, ^*∗∗*^*P* < 0.01, and ^*∗∗∗*^*P* < 0.001.

**Figure 2:** HA alleviates LPS-induced lung injury by regulating the expression of miR-204. (a) LPS treatment reduced miR-204, and HA treatment caused an upregulation of miR-204 expression; (b) miR-204 was knocked down (c) HA relieved LPS caused by regulating miR-204; (d) HA reduces the apoptosis caused by LPS by regulating miR-204; (e) HA reduces apoptosis-related proteins by regulating miR-204; (f) HA regulates miR-204 and alleviates the increase of inflammation-related factors; and (g) HA relieves the increase of inflammation-related factors by regulating miR-204. Compared with the LPS group, ^*∗*^*P* < 0.05, ^*∗∗*^*P* < 0.01, and ^*∗∗∗*^*P* < 0.001.

**Figure 3:** miR-204 targets FOXK2. (a) The targeting relationship between FOXK2 and miR-204 was verified by luciferase detection; (b) FOXK2 and miR-204 were negatively correlated. Compared with the LPS group, ^*∗*^*P* < 0.05, ^*∗∗*^*P* < 0.01, and ^*∗∗∗*^*P* < 0.001.

**Figure 4:** miR-204 participates in HA alleviating LPS-induced lung injury through targeted regulation of FOXK2. (a) Overexpression of FOXK2 in A549 cells; (b) silencing miR-204 relieves LPS-induced vitality suppression by regulating FOXK2; (c) silencing miR-204 reduces LPS-induced apoptosis by regulating FOXK2; (d) silencing miR-204 alleviates the increase in apoptosis-related protein expression caused by LPS by regulating FOXK2; (e) silencing miR-204 alleviates the increase of inflammation-related factors caused by LPS by regulating FOXK2; and (f) silencing miR-204 alleviates by regulating FOXK2 increased levels of inflammation-related factors caused by LPS. Compared with the LPS group, ^*∗*^*P* < 0.05, ^*∗∗*^*P* < 0.01, and ^*∗∗∗*^*P* < 0.001.

**Figure 5:** Silencing miR-204 inhibits the NF-*κ*B pathway by regulating FOXK2. Compared with the LPS group, ^*∗*^*P* < 0.05, ^*∗∗*^*P* < 0.01, and ^*∗∗∗*^*P* < 0.001.

## Data Availability

The simulation experiment data used to support the findings of this study are available from the corresponding author upon request.
